The article "Public Health Risk Assessment and Prevention Based on Big Data" was published in 2022. Journal: J Environ Public Health.

# Public Health Risk Assessment and Prevention Based on Big Data

**DOI:** 10.1155/2022/7965917

**Published:** 2022-09-05

**Authors:** Hua-ying Zhang, Tiande Pan

**Affiliations:** ^1^Department of Construction Information Engineering, Henan Polytechnic of Architecture, Zhengzhou 450064, China; ^2^Hezhou University School of Artificial Intelligence Hezhou City, Guangxi 542800, Zhuang Autonomous Region, China

## Abstract

In order to improve the ability of public health risk assessment in the context of community collaborative prevention and control, a mathematical model of public health risk assessment in the context of community collaborative prevention and control based on the integration and balanced allocation of big data features in the prevention horizon is proposed. The constraint parameter model of public health risk assessment under the background of community collaborative prevention and control is constructed, the method of dynamic feature analysis of joint prevention and control is adopted to realize the dynamic risk point detection of public health risk assessment data and the integration of constraint mechanism related feature points, and the fuzzy dynamic statistical feature matching method is adopted to carry out the adaptive dynamic statistics and resource balanced allocation analysis of public health risk assessment set under the background of community collaborative prevention and control. A public health risk parameter fusion model is established under the background of community collaborative prevention and control, the methods of balanced resource allocation and joint management and control are combined to realize balanced scheduling and prevention area block matching in the process of dynamic parameter estimation of public health risk evaluation data under the background of community collaborative prevention and control, the correlation distribution of public health risk under the background of community collaborative prevention and control is taken as the cost function, and balanced allocation is realized according to the statistical information sampling results of public health risk evaluation data under the background of community collaborative prevention and control. Combined with differential clustering analysis, the data clustering and attribute merging of public health risk assessment under the background of community collaborative prevention and control are realized, and the mathematical modeling optimization of public health risk assessment under the background of community collaborative prevention and control is realized. The simulation results show that this method has good adaptability, high degree of parameter fusion, and strong ability of matching risk prevention areas and balancing resource allocation in the context of community collaborative prevention and control.

The article "Public Health Risk Assessment and Prevention Based on Big Data" was published in 2022. Journal: J Environ Public Health.

## 1. Introduction

Common health risks pose a serious threat to the life, as well as health and safety of the society and people, and the harm is very serious, especially the COVID-19 epidemic situation, which makes us aware of the threat brought by public health emergencies. Therefore, speeding up the construction of early warning mechanism for public health emergencies, establishing a public health risk prevention model under the background of community collaborative control and prevention, and creating a safe and stable living and production environment are of great value to citizens' health and life safety, as well as the foundation and guarantee for promoting the harmonious development of society [1–3]. Constructing an optimized method model of public health risk under the background of community collaborative prevention and control is helpful to improve the government's ruling ability and credibility, strengthen the emergency management of public health incidents, and combine the public health risk assessment under the background of community collaborative prevention and control, which is the embodiment of people-oriented concept, the key for the government to effectively exploit its power in combination with legal provisions, and an important medium to enhance the government's credibility [4–6]. In view of public health emergencies, the government should further establish and improve the emergency management system, which will help the government to continuously improve its emergency management ability, promote the modernization of national governance system and governance ability, and establish public health risk assessment and prevention under the background of community collaborative prevention and control, which is a good proof of this aspect in promoting the emergency management and control of COVID-19 epidemic in China [2].

In short, through the establishment of public health risk assessment and prevention mechanism under the background of community collaborative prevention and control, in order to better improve the emergency treatment of public health emergencies, we should pay more attention to the emergency management of public health emergencies, strengthen the talent team, and combine big data analysis technology to build a public health risk assessment and prevention model under the background of community collaborative prevention and control. The research on related algorithms and models of public health risk assessment under the background of community collaborative prevention and control has attracted great attention [7].

The article "Public Health Risk Assessment and Prevention Based on Big Data" was published in 2022. Journal: J Environ Public Health.

It is necessary to build an optimized public health risk assessment model under the background of community collaborative prevention and control and combine the methods of risk prevention area matching and resource allocation balance control to improve the efficiency of dynamic parameter estimation of public health risk assessment data under the background of community collaborative prevention and control, so as to ensure the safety and accuracy of dynamic parameter estimation of public health risk assessment data under the background of community collaborative prevention and control. Studying the public health risk assessment model under the background of community collaborative prevention and control is of great significance to improve the security and communication stability of public health risk assessment data under the background of community collaborative prevention and control [8]. The research of public health risk assessment model under the background of community-based collaborative prevention and control has attracted great attention. In traditional methods, the public health risk assessment methods under the background of community collaborative prevention and control mainly include the public health risk assessment model based on fuzzy association rules, the public health risk assessment model based on fuzzy dynamic statistical feature matching, and the public health risk assessment method under the background of community collaborative prevention and control with balanced link control. Balanced allocation and fuzzy feature matching are adopted to achieve public health risk assessment under the background of community collaborative prevention and control, but the traditional methods have poor adaptability and weak statistical analysis ability [9].

In view of the above problems, this paper proposes a mathematical model of public health risk assessment under the background of community collaborative prevention and control based on the integration and balanced allocation of big data features from the perspective of prevention [10]. Firstly, the constraint parameter model of public health risk assessment under the background of community collaborative prevention and control is constructed, and the dynamic risk point detection of public health risk assessment data and the integration of constraint mechanism related feature points under the background of community collaborative prevention and control are realized by using the method of dynamic feature analysis of joint prevention and control, and then the public health risk parameter fusion model under the background of community collaborative prevention and control is established. Combining the methods of balanced resource allocation and joint management and control, the balanced scheduling and the matching of prevention areas in the process of dynamic parameter estimation of public health risk evaluation data under the background of community collaborative prevention and control are realized. Taking the correlation distribution of public health risk under the background of community collaborative prevention and control as the cost function, the balanced allocation of transmission efficiency is realized according to the statistical information sampling results of public health risk evaluation data under the background of community collaborative prevention and control, and the clustering and attribute merging of public health risk evaluation data under the background of community collaborative prevention and control are combined with the method of differential clustering analysis, so that the mathematical modeling optimization of public health risk evaluation under the background of community collaborative prevention and control is realized. Finally, the simulation test shows that this method has superior performance in improving the accuracy and balance of public health risk assessment under the background of community collaborative prevention and control.

The article "Public Health Risk Assessment and Prevention Based on Big Data" was published in 2022. Journal: J Environ Public Health.

## 2. Constraint Parameters and Balanced Control of Public Health Risks in the Context of Community Collaborative Prevention and Control

At present, the research characteristics of risk assessment of public health emergencies at home and abroad are mainly reflected in the following aspects:

1. Major Infectious Diseases
2. This kind of risk assessment tends to cover the comprehensive evaluation of biology, sociology, and economics. Based on historical data and field investigation, most of the existing studies have established a risk assessment index system through Delphi method, brainstorming method, expert scoring method, and so forth, determined the index weight, and established a comprehensive evaluation model of disease occurrence risk by using comprehensive scoring method or analytic hierarchy process.
3. Acute Physical and Chemical Exposure
4. This kind of research involves the types, physical and chemical properties, existing forms, exposure time, and exposure concentration of dangerous goods. It mostly adopts the combination of qualitative and quantitative analysis for risk assessment. Some scholars use data mining technology and fuzzy neural network to carry out the risk assessment research of acute physical and chemical exposure.
5. Food-Borne Diseases
6. This kind of risk assessment mostly collects sufficient information through epidemiological research, toxicological research, in vitro experiments, and so forth and establishes models of exposure dose and adverse reactions so as to estimate the possible adverse effects of people exposed to a specific risk source and put forward corresponding risk response strategies. Quantitative microbial risk assessment is the main method of food-borne disease risk assessment. It mainly simulates the possibility of pathogenic bacteria infection caused by food consumption in the food chain, determines the countermeasures that can be taken in the food chain, and evaluates the effects of various measures.
7. Major Events
8. This kind of risk assessment is mainly to identify all risks and their characteristics that may exist in a certain period of time and in a certain area. This kind of research mostly adopts the risk matrix method.

The article "Public Health Risk Assessment and Prevention Based on Big Data" was published in 2022. Journal: J Environ Public Health.

### 2.1. Constraint Parameters of Public Health Risk in the Context of Community Collaborative Prevention and Control

In order to realize the public health risk assessment under the background of community collaborative prevention and control, the constraint parameter model of public health risk assessment under the background of community collaborative prevention and control is constructed. The quantitative equilibrium scheduling model of public health risk assessment data under the background of community collaborative prevention and control is constructed by using the method of spatial equilibrium control, and the constraint parameter model of public health risk assessment under the background of community collaborative prevention and control is constructed [11]. The dynamic risk point detection of public health risk assessment data under the background of community collaborative prevention and control and the integration of constraint mechanism related feature points are realized by using the method of joint prevention and control dynamic feature analysis. The fuzzy clustering state parameter of public health risk evaluation data under the background of community collaborative prevention and control is *T*=Δ*L* · *L*_*m*_. Firstly, a distributed data storage structure model of public health risk index distribution big data under the background of community collaborative prevention and control is constructed, and a quadruple G is used to represent the storage distribution structure of public health risk index distribution big data under the background of community collaborative prevention and control, which is *c*, assuming that it is the detection dimension of public health risk index distribution big data under the background of community collaborative prevention and control, and *W*_*ij*_^(*K*)^ represents the number of public health risk evaluation distribution sets under the background of community collaborative prevention and control. It represents the activity of the first node in the data sampling of public health risk index distribution big data in the context of *i* community collaborative prevention and control, extracts the correlation matching feature quantity of public health risk index distribution big data in the context of community collaborative prevention and control, and adopts multidimensional information scheduling, in which *F*^2*α*/*π*^=∑_*i*=0_^3^*a*_*i*_(*α*)*W*^*i*^, combined with fuzzy detection method, establishing the feature distribution set of public health risk evaluation data in the context of community collaborative prevention and control. Based on big data analysis technology and discrete scheduling method [12], the grid distribution model is shown in Figure 1.

The article "Public Health Risk Assessment and Prevention Based on Big Data" was published in 2022. Journal: J Environ Public Health.

Furthermore, the conditions for stable transmission of parameters of the diversity model of public health risk evaluation data under the background of community collaborative prevention and control are expressed in the following formula:

(1) $$\begin{array}{c} 0<\Delta L<1+\frac{\lambda_{2}}{L}, \end{array}$$

where *L* is the dynamic parameter of public health risk indicators under the background of community collaborative prevention and control and *λ* is the ambiguity coefficient. By adopting the method of full data set fusion, the efficiency evaluation model of dynamic parameter estimation of public health risk evaluation data under the background of community collaborative prevention and control is established [13], and the regression analysis model of public health risk under the background of community collaborative prevention and control is established by combining the methods of expert feedback and pattern recognition, and the risk prevention area block matching and resource allocation equilibrium control model of dynamic parameter estimation of public health risk evaluation data under the background of community collaborative prevention and control are obtained. Setting *∂π*_*m*_/*∂p*_1_=0, *∂π*_*m*_/*∂A*_1_=0, and *η*=2*μ*_2_*δ*(1 − *δ*) − *ρ*_2_^2^, the expression of risk prevention area block matching and resource allocation equilibrium control parameter model for dynamic parameter estimation of public health risk evaluation data under the background of community collaborative prevention and control is as follows:

(2) $$\begin{array}{c} \frac{2\delta^{2}\left(1-\delta \right)\mu_{2}-2\rho_{2}^{2}\delta -2\eta }{\left(1-\delta \right)\eta }p_{1}\\ +\frac{\rho_{1}\cdot \rho_{2}^{2}\delta \left(1-\delta \right)-\left(1-\delta \right)\delta \mu_{2}\rho_{1}+\rho_{1}\eta }{\left(1-\delta \right)\eta }A_{1}\\ +Q+\frac{\delta \left(1-\delta \right)\mu_{2}\left[\delta \left(1-\delta \right)\mu_{2}-2\rho_{2}^{2}\right]+\rho_{2}^{2}\left(\eta +\rho_{2}^{2}\right)}{\delta {\left(1-\delta \right)}^{2}\mu_{2}\eta }\left(c_{2}+c_{r}\right)\\ -\frac{\delta^{2}\left(1-\delta \right)\mu_{2}-\delta \rho_{2}^{2}-\eta }{\left(1-\delta \right)\eta }c_{2}=0, \end{array}$$

where *ρ*_1_ and *ρ*_2_ are the clustering centers of public health risk index distribution big data under the background of community collaborative prevention and control, *A*_1_ is the sample amplitude of public health risk index distribution big data, *p*_1_ is the statistical characteristic quantity, *Q* is the correlation coefficient, *η* is the ambiguity, and *δ* is the similarity coefficient. On the global outlier data set, combined with the ambiguity parameter identification method [14], a density grid cluster center classification set of dynamic parameter estimation of public health risk evaluation data under the background of community collaborative prevention and control is established, and the grid partition block matching by fuzzy parameter identification of data in grid object is realized. The efficiency regression analysis value of dynamic parameter estimation of public health risk evaluation data under the background of community collaborative prevention and control satisfies *e*^−*L*_*m*_*s*^=1 − *L*_*m*_*s*. Under the grid clustering model of two-dimensional data sets, the grid clustering results are as follows:

(3) $$\begin{array}{c} g_{\alpha }^{\prime }\left(u\right)=A_{\alpha }\int_{-\infty }^{+\infty }\exp\left[j{\left(u-t\right)}^{2}\csc\alpha \right]g\left(t\right)dt, \end{array}$$

where *g*(*t*) is the cost function of public health risk constraint under the background of community collaborative prevention and control, *h*(*u* − *t*) is the density value of each risk control grid object, and *A*_*α*_ is the deep fusion characteristic value of public health risk index distribution big data under the background of community collaborative prevention and control. The probability density *y*_*s*_ of *w*_*s*_*s* is calculated by *X*_*p*_(*u*), the characteristic sampling interval of public health risk evaluation data under the background of community collaborative prevention and control is *A*_*α*_, and the stable characteristic solution with cluster center is automatically determined as in the two following formulas:

(4) $$\begin{array}{c} Ε\left[{\tilde{e}}_{sk}\right]=0,\;\forall s=1,\ldots ,n,\;k=1,\ldots ,p, \end{array}$$

(5) $$\begin{array}{c} Ε\left[{\tilde{e}}_{s1k1}{\tilde{e}}_{s2k2}\right]=\left\{\begin{array}{c} \frac{m}{p}\sigma_{s}^{2},\\ 0. \end{array}\right. \end{array}$$

In the above formulas, *s* is the fuzzy closeness between big data sharing nodes, *σ*_*s*_^2^ is matching feature, *p* is the error, and *m* is the embedding dimension; *α*, *β*, *γ*, and *ρ* are the standardized residual learning cost factors; *D*(*c*) ≡ *c*^*d*^mod*n* ≡ (*m*^*e*^)^*d*^mod*n*; it can be known that the constraint cost function is stable and convergent. The dynamic feature analysis method of prevention and joint control is adopted to realize the dynamic risk point detection of public health risk evaluation data under the background of community collaborative prevention and control and the integration of constraint mechanism related feature points, so as to improve the public health risk evaluation data under the background of community collaborative prevention and control [15].

The article "Public Health Risk Assessment and Prevention Based on Big Data" was published in 2022. Journal: J Environ Public Health.

### 2.2. Clustering Analysis of Public Health Risk Evaluation Data Fusion

Fuzzy dynamic statistical feature matching method has the advantages of good data fusion effect and fast fusion speed. The basic idea of fuzzy matching is to calculate the similarity between each string and the target string and take the string with the highest similarity as the fuzzy matching result with the target string. For calculating the similarity between strings, the most common idea is to use the edit distance algorithm. The steps of the algorithm are as follows:

Construct a matrix with rows of *m*+1 and columns of *n*+1, which is used to save the number of operations required to complete a conversion, and the number of operations required to convert the string *s*[1 … *N*] to the string *t*[1 … *M*] is the value of matrix [*n*][*m*].
Initialize the first row of matrix from 0 to *N* and the first column from 0 to *M*.
Check each *s*[*i*] character from 1 to *N*.
Check each *s*[*i*] character from 1 to *m*.
Compare each character of string *s* and string *t* in pairs. If they are equal, let cost be 0; if they are not equal, let cost be 1 (this cost will be used later).
(a) If we can convert *s*[1 … *I* − 1] into *t*[1 … *J*] in *K* operations, we can remove *s*[*i*] and then do these *K* operations, so a total of *k*+1 operations are required. (b) If we can convert *s*[1 … *I*] into *t*[1 … *J* − 1] within *K* operations, that is, *d*[*i*,  *j* − 1]=*k*, then we can add *t*[*j*] and *s*[1 … *I*], so a total of *k*+1 operations are required. (c) If we can convert *s*[1 … *I* − 1] into *t*[1 … *J* − 1] in *K* steps, we can convert *s*[*i*] into *t*[*j*], so that *s*[1 … *I*]==*t*[1 … *J*], which also requires *k*+1 operations in total (cost is added here because if *s*[*i*] is just equal to *t*[*j*], then there is no need to do another replacement operation, which can be satisfied; if it is not equal, there is a need to do another replacement operation, which requires *k*+1 operations). (d) Repeat 3, 4, 5, and 6, and the final result is in *d*[*n*, *m*].

The article "Public Health Risk Assessment and Prevention Based on Big Data" was published in 2022. Journal: J Environ Public Health.

Fuzzy dynamic statistical feature matching method is used to analyze the adaptive dynamic statistics and resource balance allocation of public health risk assessment set under the background of community collaborative prevention and control. By fitting data points, the fuzzy parameters of dynamic parameter estimation of public health risk assessment data under the background of community collaborative prevention and control are *K*_*b*_^*bw*^(*S*), *K*_*d*_^*cp*^(*S*), *D*_*a*,*p*_, and *Mα*_*a*,*b*_. Combined with multipath time delay compensation method, the spatial fusion clustering and feature sampling of discrete time series of public health risk assessment data under the background of community collaborative prevention and control are completed by residual analysis, and the distribution concept set of public health risk assessment data under the background of community collaborative prevention and control is obtained as follows:

(6) $$\begin{array}{c} F_{\alpha }\left[e^{j\pi \left(2f_{0}t+k_{0}t^{2}\right)}\right]=\sqrt{\frac{1+i\tan\alpha }{1+k_{0}\tan\alpha }}\times \exp\left[i\pi \frac{u^{2}\left(k_{0}-\tan\alpha \right)+2uf_{0}\sec\alpha -f_{0}\tan\alpha }{1+k_{0}\tan\alpha }\right], \end{array}$$

where *G*_*α*_ is the connected finite graph of the distribution of public health risk indicators in the context of community collaborative prevention and control, *u* is the marginal feature quantity, *f*_0_ is the risk prevention subspace, *α* is the sampling frequency spectrum, *k*_0_ is the normalized distribution error of big data of public health risk indicators in the context of community collaborative prevention and control, and *α* − arctg(*k*_0_)=(2*j*+1/2)*π* is the regression distribution set. In the fitting decision graph, a density grid distribution model of dynamic parameter estimation of public health risk evaluation data in the context of community collaborative prevention and control is as follows:

(7) $$\begin{array}{c} F_{\alpha }=\sqrt{\frac{1}{\left(1-ik_{0}\right)}}\delta \left(u-f_{0}\sin\alpha \right), \end{array}$$

where *k*_0_ is the recursive coefficient of public health risk assessment under the background of community collaborative prevention and control. Combined with the fuzzy optimization method and the standardized residual analysis method, the data fusion cluster analysis of public health risk assessment under the background of community collaborative prevention and control is realized [16–18].

The article "Public Health Risk Assessment and Prevention Based on Big Data" was published in 2022. Journal: J Environ Public Health.

## 3. Optimization of Public Health Risk Assessment under the Background of Community Collaborative Prevention and Control

### 3.1. Community Collaborative Prevention and Control in the Context of Public Health Risk Assessment Data Dynamic Parameter Estimation Balanced Scheduling

Combining the methods of balanced resource allocation and joint management and control to realize balanced scheduling and matching of prevention areas in the process of dynamic parameter estimation of public health risk evaluation data under the background of community collaborative prevention and control [19, 20], taking the correlation distribution of public health risks under the background of community collaborative prevention and control as the cost function, making *F* the limited domain of dynamic parameter estimation of public health risk evaluation data under the background of community collaborative prevention and control, it is the multipath characteristic component of public health risk evaluation data under the background of community collaborative prevention and control [21]. In the balanced allocation model of risk prevention area block matching and resource allocation, the common marker characteristic set of *H*2 and *H*3 is *X*. If *A*=(*a*_*i*,*j*_)_*i*,*j*=1_^*m*^ and *B*=(*b*_*i*,*j*_)_*i*,*j*=1_^*m*^ are used to fit the data points, the linear fitting model of public health risk evaluation data under the background of community collaborative prevention and control is as follows:

(8) $$\begin{array}{c} \text{State}\left(K,N\right)0=-\mu p_{k,N}+\lambda p_{K-1,N}+rp_{K,N-1}, \end{array}$$

where *μ* is the partition size of risk management and control and *p*_*k*,*N*_ is the size of resource allocation grid. The fuzzy dynamic statistical feature matching method is used to analyze the adaptive dynamic statistics and resource balance allocation of public health risk assessment set under the background of community collaborative prevention and control, and the fusion model of public health risk parameters under the background of community collaborative prevention and control is established. Combining the methods of balanced resource allocation and joint management and control, the balanced scheduling and the matching of prevention areas in the process of dynamic parameter estimation of public health risk evaluation data under the background of community collaborative prevention and control are realized. In the process of resource allocation, the fuzzy identification parameter model of dynamic parameter estimation of public health risk evaluation data under the background of community collaborative prevention and control is obtained by using the method of two-dimensional data set planning. In the normalized residual diagram *Q*, the inverse matrix *Q*^−1^ is obtained, and the binary transformation of *Q*^−1^ is performed, and the intervariable function of public health risk estimation under the background of community collaborative prevention and control is as follows:

(9) $$\begin{array}{c} \left\{\begin{array}{c} Q_{1}\left(s\right)=M_{-}^{-1}\left(s\right)f_{1}\left(s\right),\\ Q_{2}\left(s\right)=M_{-}^{-1}\left(s\right)f_{2}\left(s\right), \end{array}\right. \end{array}$$

where *f*_1_(*s*) is the characteristic vector of public health risk index distribution big data under the background of community collaborative prevention and control, *f*_2_(*s*) is the joint correlation distribution set, and *M*_−_^−1^(*s*) is the grid block coefficient. If *e*_*st*1_ is independent of *e*_*st*2_, the high-precision fitting model of public health risk planning under the background of noncommunity collaborative prevention and control is as follows:

(10) $$\begin{array}{c} \left\{\begin{array}{c} C_{1}\left(s\right)=\frac{\lambda_{2}s+1}{\lambda_{1}s+1},\\ C_{2}\left(s\right)=\frac{\prod_{i=1}^{i=n}\left(T_{mi}s+1\right)}{K_{m}\left(\lambda_{2}+L_{m}\right)s} \end{array}\right., \end{array}$$

where *T*_*mi*_ is the connected graph structure of health risk index distribution, *s* is the sampling characteristic point, and *L*_*m*_ is the fuzziness of big data of public health risk index distribution under the background of district collaborative prevention and control. In the nearest neighbor direction, the characteristic solutions of decision optimization matrix and convergence matrix of dynamic parameter estimation equilibrium configuration function of public health risk evaluation data under the background of community collaborative prevention and control are obtained. In summary, the balanced scheduling and efficiency evaluation of dynamic parameter estimation of public health risk evaluation data under the background of community collaborative prevention and control are realized, and the fusion cluster analysis is carried out according to the efficiency evaluation results [22].

The article "Public Health Risk Assessment and Prevention Based on Big Data" was published in 2022. Journal: J Environ Public Health.

### 3.2. Mathematical Model of Public Health Risk Assessment under the Background of Community Collaborative Prevention and Control

In the process of building the mathematical model of public health risk assessment, based on the statistical information sampling results of the above public health risk assessment data, the big data method is used to establish it. Big data technology refers to the application technology of big data, covering all kinds of big data platforms, big data index system, and other big data application technologies. Big data refers to data sets that cannot be captured, managed, and processed by conventional software tools within a certain time range. A bilevel programming hyperbolic model for dynamic parameter estimation of public health risk evaluation data in the context of community collaborative prevention and control is obtained, as shown in the following formula:

(11) $$\begin{array}{c} \left\{\begin{array}{c} u_{tt}-\Delta u+{\left|u\right|}^{4}cu=0,\\ {\left(u,\partial_{t}u\right)|}_{t=0}=\left(u_{0},u_{1}\right)\in {\dot{H}}_{x}^{s_{c}}\times {\dot{H}}_{x}^{s_{c}-1}, \end{array}\right. \end{array}$$

where the adjacent grid size is Δ*u*, *u* is the search radius, and ${\dot{H}}_{x}^{s_{c}}$ is the parameter fitness; it can get the characteristic points of public health risk evaluation data under the background of community collaborative prevention and control. Combined with the dynamic parameter estimation of public health risk evaluation data under the background of community collaborative prevention and control and the distance estimation method of nonedge points of risk prevention area block matching and resource allocation, the steady characteristic solution *β* = (*β*_1_, ⋯,*β*_*m*_)^*T*^ ∈ *GF*(2^*n*^)^*m*^ is obtained, and the stable periodic solution of public health risk evaluation under the background of community collaborative prevention and control is obtained by dichotomy as follows: combining the gridding results of 2D data sets to complete feature decomposition, the output is

(12) $$\begin{array}{c} F^{p}=\exp\left(j\pi \rho^{2}\sin\alpha \cos\alpha \right), \end{array}$$

where *ρ* is the identification degree of public health risk assessment under the background of community collaborative prevention and *α* is the quantitative parameter allocation set. By using the finite dimensional analysis method, the reliability function of public health risk assessment under the background of community collaborative prevention and control is expressed by *s*^*∗*^ = {*x* ∈ *X|f*(*x*) = max*f*(*x*)}. According to the best game state parameters of public health risks obtained in the context of community collaborative prevention and control, the characteristic data of public health risk assessment in the context of community collaborative prevention and control is obtained, which satisfies formula as follows:

(13) $$\begin{array}{c} f\left(x_{1}\right)=f\left(x_{2}\right)=\cdots =f\left(x_{n}\right)=f^{*}, \end{array}$$

where *f*(*x*_1_),…… *f*(*x*_*n*_) are the blockchain fusion functions of public health risk management. According to the above analysis, the big data fusion scheduling of public health risk assessment under the background of community collaborative prevention and control is realized, and the fitting value *Y*^*∗*^ of response variable *Y* is obtained, so that *I* = {*i|* ≤ *s*_*i*_ ≥ *s*_*j*_, ∀*s*_*j*_ ∈ *S*^1^} can meet the statistical characteristics of public health risk under the background of community collaborative prevention and control [23].

The article "Public Health Risk Assessment and Prevention Based on Big Data" was published in 2022. Journal: J Environ Public Health.

According to the corresponding observation values and fitting values, the clustering and attribute merging of public health risk evaluation data under the background of community collaborative prevention and control are realized by using the method of fusion differential clustering analysis, and the mathematical modeling optimization of public health risk evaluation under the background of community collaborative prevention and control is realized. The linear fitting results of dynamic parameter estimation and evaluation of public health risk evaluation data under the background of community collaborative prevention and control are as follows:

(14) $$\begin{array}{c} p_{id}^{new}=\left\{\begin{array}{cc} p_{id}+m\left(\right)\left(X_{\max}-p_{id}\right), & if\;m\left(\right)>0,\\ p_{id}+m\left(\right)\left(p_{id}-X_{\min}\right), & if\;m\left(\right)\leq 0, \end{array}\right. \end{array}$$

where *X*_max_ and *X*_min_ are the maximum threshold and the minimum threshold, respectively, and *p*_*id*_ is the probability density of public health risk assessment. To sum up, we can realize the optimal design of the mathematical model of public health risk assessment under the background of community collaborative prevention and control. To sum up, taking the correlation distribution of public health risks in the context of community collaborative prevention and control as the cost function, the balanced allocation of transmission efficiency is realized according to the statistical information sampling results of public health risk assessment data in the context of community collaborative prevention and control, and the clustering and attribute merging of public health risk assessment data in the context of community collaborative prevention and control are realized by combining the fusion differential cluster analysis method, thus realizing the mathematical modeling optimization of public health risk assessment in the context of community collaborative prevention and control [21, 24]. The realization process is shown in Figure 2.

## 4. Simulation Test

In the simulation test of public health risk assessment under the background of community collaborative prevention and control, the scale of public health risk assessment data under the background of community collaborative prevention and control is set to be 1200 Mbit, the number of iterations of assessment is 200, the prior probability density of public health risk assessment under the background of community collaborative prevention and control is 0.55, the correlation coefficient of public health risk assessment under the background of community collaborative prevention and control is 0.103, and the adaptive weighting coefficient is 0.14. The distribution of the optimized coordinate system of public health risk management and control under the background of community collaborative prevention and control is shown in Figure 3.

The article "Public Health Risk Assessment and Prevention Based on Big Data" was published in 2022. Journal: J Environ Public Health.

Dynamic feature analysis of joint prevention and control is used to realize the dynamic risk point detection of public health risk evaluation data under the background of community collaborative prevention and control and the integration of constraint mechanism related feature points. The variable distribution of public health risk evaluation under the background of community collaborative prevention and control is shown in Table 1.

According to the above parameter settings, the public health risk assessment model under the background of community collaborative prevention and control is constructed, and the block matching results of public health risk assessment are shown in Table 2.

According to the above data analysis results, the risk assessment is realized, and the distribution of public health risk assessment data under the background of community collaborative prevention and control is shown in Figure 4.

According to the distribution characteristics of public health risk evaluation data under the background of community collaborative prevention and control in Figure 4, the public health risk evaluation under the background of community collaborative prevention and control is realized, and the scattered distribution diagram of dynamic parameter estimation of public health risk evaluation data under the background of community collaborative prevention and control is shown in Figure 5.

According to the scattered distribution diagram of dynamic parameter estimation of public health risk evaluation data under the background of community collaborative prevention and control in Figure 5, the convergence judgment of public health risk under the background of community collaborative prevention and control is realized, and the results are shown in Figure 6.

From the analysis of Figure 6, it can be seen that the convergence of this method in public health risk assessment under the background of community collaborative prevention and control is good. The accuracy of the evaluation is shown in Table 3, and the comparison results show that the accuracy of public health risk assessment is high under the background of community collaborative prevention and control.

The article "Public Health Risk Assessment and Prevention Based on Big Data" was published in 2022. Journal: J Environ Public Health.

In order to further test the reliability of this algorithm for public health risk assessment, the assessment accuracy of the four characteristic nodes in public health risk assessment using this algorithm is counted, and the statistical results are shown in Figure 7.

According to the results in Figure 7, we can see that the accuracy of using this algorithm to evaluate the probability of public health risk is more than 65%, which shows that this algorithm not only can effectively evaluate the probability of public health risk but also has a high evaluation accuracy. This is because this algorithm is based on the reliability index of evaluating the probability of public health risk. The fuzzy dynamic statistical feature matching method is used to obtain all subnodes of the reliability index state vector, and the mathematical model of big data risk assessment is constructed to achieve high-accuracy assessment.

On this basis, compare the methods of literature [2] and literature [3] to calculate the computational complexity of the proposed algorithm. The shorter the time of the algorithm, the lower the computational complexity. Therefore, the experiment was carried out with the evaluation time as the test index, and the experimental results are shown in Figure 8.

As shown in Figure 8, under the same conditions, the proposed method takes the shortest time, indicating that the proposed method has the lowest computational complexity, the strongest operability, and high practical applicability.

## 5. Conclusions

In order to optimize the performance of public health risk assessment, this paper proposes a public health risk assessment and prevention research based on big data. On the basis of clarifying the public health risk constraint parameters, a mathematical model of public health risk assessment based on feature fusion and balanced allocation of correlated big data is constructed. The analysis shows that, after the application of this method, the accuracy of public health risk assessment is high and the convergence is good.

## Figures and Tables

**Figure 1:** Public health risk control grid under the background of community collaborative prevention and control.

**Figure 2:** Implementation process of public health risk management and control under the background of community collaborative prevention and control.

**Figure 3:** Optimized coordinate system of public health risk control under the background of community collaborative prevention and control.

**Figure 4:** Public health risk evaluation data under the background of community collaborative prevention and control.

The article "Public Health Risk Assessment and Prevention Based on Big Data" was published in 2022. Journal: J Environ Public Health.

**Figure 5:** Scattered distribution of dynamic parameter estimation of public health risk evaluation data under the background of community collaborative prevention and control.

**Figure 6:** Convergence judgment of public health risk under the background of community collaborative prevention and control.

**Figure 7:** Evaluation accuracy.

**Figure 8:** Comparison of evaluation time of different methods.

**Table 1:** Variable distribution of public health risk assessment in the context of community collaborative prevention and control.

Variable	Mean value	Standard value	Minimum value	Statistical value
Similarity	0.830	0.7410	4.759	12.252
Degree of association	0.571	0.0884	4.594	12.817
Proportionality	0.413	0.9692	4.980	12.165
Reliability	0.113	0.9214	4.930	12.932
Ambiguity coefficient	0.467	0.2085	4.801	12.952
Regression analysis value	0.468	0.2383	4.931	12.703

**Table 2:** Block matching results of public health risk assessment.

Evaluation area	Statistical sample number	Reliability factor	Fuzzy kernel coefficient	Information entropy
1	9429	0.895	17.060	6.304
2	8756	0.961	9.006	4.026
3	5597	0.088	4.264	3.791
4	2461	0.308	8.997	7.256
5	7290	0.468	3.346	4.632
6	7694	0.820	4.780	9.172
7	9133	0.538	7.114	7.237
8	3007	0.136	7.548	6.820
9	8128	0.370	1.483	3.134
10	7176	0.457	5.028	9.184
11	6516	0.400	0.742	2.983
12	4207	0.633	6.189	0.520

**Table 3:** Accuracy test of public health risk assessment under the background of community collaborative prevention and control.

Iterations	This method	Statistical analysis	Fuzzy degree identification
100	0.942	0.821	0.814
200	0.965	0.854	0.832
300	0.991	0.904	0.854
400	0.995	0.924	0.914

## Data Availability

The raw data supporting the conclusions of this article will be made available by the authors, without undue reservation.
